# Identification of Candidate MicroRNA-mRNA Subnetwork for Predicting the Osteosarcoma Progression by Bioinformatics Analysis

**DOI:** 10.1155/2022/1821233

**Published:** 2022-09-22

**Authors:** Dejie Lu, Hanji Huang, Li Zheng, Kanglu Li, Xiaofei Cui, Xiong Qin, Mingjun Zheng, Nanchang Huang, Chaotao Chen, Jinmin Zhao, Bo Zhu

**Affiliations:** ^1^Guangxi Engineering Center in Biomedical Materials for Tissue and Organ Regeneration, The First Affiliated Hospital of Guangxi Medical University, Nanning 530021, China; ^2^Collaborative Innovation Centre of Regenerative Medicine and Medical BioResource Development and Application Co-constructed by the Province and Ministry, Guangxi Medical University, Nanning 530021, China; ^3^Department of Orthopedics Trauma and Hand Surgery, The First Affiliated Hospital of Guangxi Medical University, Nanning 530021, China; ^4^International Joint Laboratory of Ministry of Education for Regeneration of Bone and Soft Tissues, The First Affiliated Hospital of Guangxi Medical University, Nanning 530021, China; ^5^Department of Bone and Soft Tissue Surgery, Guangxi Medical University Cancer Hospital, Nanning 530021, China; ^6^Guangxi Key laboratory of Regenerative Medicine, The First Affiliated Hospital of Guangxi Medical University, Nanning 530021, China

## Abstract

Osteosarcoma (OS) is the pretty common primary cancer of the bone among the malignancies in adolescents. A single molecular component or a limited number of molecules is insufficient as a predictive biomarker of OS progression. Hence, it is necessary to find novel network biomarkers to improve the prediction and therapeutic effect for OS. Here, we identified 230 DE-miRNAs and 821 DE-mRNAs through two miRNA expression-profiling datasets and three mRNA expression-profiling datasets. We found that hsa-miR-494 is closely linked with the survival of OS patients. In addition, we analyzed GO and KEGG enrichment for targets of hsa-miR-494-5p and hsa-miR-494-3p through R programming. And five mRNAs were predicted as common targets of hsa-miR-494-5p and hsa-miR-494-3p. We further revealed that upregulated TRPS1 was strongly correlated with poor outcomes in OS patients through the survival analysis based on the TARGET database. The qRT-PCR study verified that the expression of hsa-miR-494-5p and hsa-miR-494-3p was declined considerably, while TRPS1 was notably raised in OS cells when compared to the osteoblasts. Thus, we generated a new regulatory subnetwork of key miRNAs and target mRNAs using Cytoscape software. These results indicate that the novel miRNA-mRNA subnetwork composed of hsa-miR-494-5p, hsa-miR-494-3p, and TRPS1 might be a characteristic molecule for assessing the prognostic value of OS patients.

## 1. Introduction

Osteosarcoma (OS) is the primary cancer of the bone that arises in young teenagers [1]. According to reports, this disorder has become the second primary reason for tumor-associated deaths in adolescents [2]. Approximately one to three out of every million people suffer from this disease every year globally, and lung metastases are the prominent reason of death [3]. The current treatment for the primary tumor in patients with OS is adjuvant medication, surgery, and radiation therapy. Regrettably, these treatments often fail to get rid of cancer altogether, and it still frequently recurs and metastasizes even after the above treatment, resulting in a high mortality rate [4]. Early diagnosis of OS is tricky because the disease lacks a sensitive diagnostic marker to monitor the condition early and predict the prognosis of patients. Hence, it is a substantial unmet need to identify a new and accurate biomarker unique to OS to improve the diagnosis and prognosis of OS.

MicroRNAs (miRNAs) have been proven to be one of the most common endogenous noncoding RNAs, which can bind to the 3′ noncoding sequence of particular messenger RNAs (mRNAs) to modulate their translational performance and stability [5]. Recently, a good deal of investigations has indicated that abnormal changes of miRNAs partake in the regulation of the occurrence and development of different types of human malignancies and are associated with cell development, cell proliferation, apoptosis, and tumorigenesis [6–8]. Thus, miRNAs are considered to be outstanding biomarkers for the diagnostic analysis, targeting therapy, and prediction of malignant tumors. Nowadays, increasing researches have elucidated that miRNAs are strongly related to the carcinogenesis of OS. The differentially expressed miRNAs negatively regulate the expression level of target mRNA, providing new clues for the early diagnosis, clinical precision therapy, and prognosis evaluation of OS. For instance, hsa-miR-124 and hsa-miR-101 levels were remarkably reduced in serum from patients with OS. These two lowly expressed miRNAs were positively related to clinical progression or metastasis of lung of OS. These OS patients with a highly expressed hsa-miR-124 or hsa-miR-101 had more prolonged overall survival and better prognoses [9, 10]. In addition, hsa-miR-21, hsa-miR-221, and hsa-miR-106a have been discovered to be significantly increased in the circulating blood of patients with OS, and their alteration is tightly related to the differentiated degree, stage of neoplastic lesions, and pulmonary metastasis of OS [11]. Although many researchers are committed to establishing miRNA-based prognostic and diagnostic biomarkers in OS and have achieved outstanding results, most attention to OS biomarker prediction is indulged in single or limited miRNAs. Therefore, the clinical application of the recognized miRNAs as predicted markers of OS remains limited by the lack of specific and sensitive regulatory networks.

The thermodynamic stability of the miRNA-mRNA interaction has been demonstrated to be necessary for modulating the potential targets [12]. Thus, understanding the interaction of miRNA and mRNA expression patterns during the development of OS is of positive significance for revealing the molecular regulation mechanisms and prognostic markers of OS. The regulation of miRNA-mRNA interaction networks has been widely explored in many malignancies. Wang et al. [13] discovered three significantly associated miRNA-mRNA pairs in colorectal cancer, and the correlation of these networks with MSI and CIN signaling pathways, which is of great help to the diagnosis and healing of colorectal cancer. A novel miRNA-mRNA regulatory biomodule has been identified in human prostate cancer [14]. Wang et al. [15] also generated a potentially functional regulatory network composed of miRNA and mRNA in lung adenocarcinoma (LUAD) using bioinformatics technology. They explored the potential functions of hub miRNAs and mRNAs in this regulatory network, which will contribute to identifying novel predictive biomarkers and promote molecular targeting therapy for the patients with LUAD in clinical. These findings indicated that the regulatory networks consisting of miRNAs and mRNAs have critical functions in the tumorigenesis and progression of malignant illnesses. However, the whole picture of the miRNA-mRNA regulation network and their precise mechanisms and specificity in OS have not yet been fully revealed.

In our study, we conducted compositive bioinformatics analyses to explore the biological functions of miRNA with survival significance in OS, canonical pathways of target genes, and screening of key target mRNAs. We successfully identified predictive miRNA-target gene regulatory network patterns and functional candidate miRNA-mRNA pairs related to the tumorigenesis and prognosis of OS, thereby establishing a new miRNA-mRNA regulatory subnetwork for OS. Our findings expanded the knowledge of the tumor biology of OS by revealing a new miRNA-mRNA network landscape, which may offer valuable diagnostic markers and molecular therapeutic targets for OS.

## 2. Methods

### 2.1. Data Obtaining and Processing

To explore miRNA-mRNA regulatory networks that may affect the occurrence and development of OS, we downloaded two preprocessed miRNA microarray datasets (GSE79181 and GSE28425) and three preprocessed mRNA microarray datasets (GSE16091, GSE16088, and GSE14359) from the online database, Gene Expression Omnibus (GEO). The GSE79181 dataset contained 25 OS samples with complete clinical survival information. The GSE28425 dataset contained 19 OS tissues and 4 normal tissues without clinical information. In addition, to avoid sample heterogeneity errors caused by different platforms of technology and different ways of data processing when analyzing a more significant number of samples, these three mRNA datasets (GSE16091, GSE16088, and GSE14359) were merged and normalized using the “SVA” package in R. And all information on OS samples is exhibited in Table 1. The detailed workflow of this research is illustrated with a diagram (Figure 1).

### 2.2. Screening for Key miRNAs

The “limma” package was adopted in R to pick up differentially expressed miRNAs (DE-miRNAs) between OS specimens and matched standard specimens from GSE28425. While a package of survival analysis, “survival,” was utilized to perform a batch survival analysis from GSE79181. The candidate miRNAs were obtained from the intersection of miRNAs with survival significance and DE-miRNAs, showing in a Venn diagram through Venny2.1.

### 2.3. Screening for Key mRNAs

The same method as that used to analyze DE-miRNAs was used to gain differentially expressed mRNAs (DE-mRNAs) from the merged mRNA dataset. The mRNAs with a threshold value of *p* value is less than 0.05, as well as log2(fold − change) > 1 or log2(fold − change) < −1, were known as DE-mRNAs. In addition, four online prediction databases, miRWalk (http://mirwalk.umm.uni-heidelberg.de/), RNAhybrid (https://bibiserv.cebitec.uni-bielefeld.de/rnahybrid/), Targetscan (http://www.targetscan.org/vert_71/), and miRanda (http://www.microrna.org/microrna/home.do), were employed to forecast the potential targeting mRNAs of candidate miRNAs. The candidate mRNAs were obtained by intersecting the predicted target mRNAs with DE-mRNAs.

### 2.4. Investigation of Gene Ontology and Kyoto Encyclopedia of Genes and Genomes

To explore the molecular roles of key miRNAs' target genes, the enrichment investigations of the Gene Ontology (GO) and Kyoto Encyclopedia of Genes and Genomes (KEGG) were achieved via utilizing the “clusterProfiler” package in R [16]. Additionally, the “ggplot2” package was used to visualize better the connection between candidate genes and classical biological function and signaling pathway.

### 2.5. Generation of miRNA-mRNA Regulation Subnetwork

The regulation network composed of miRNAs and particular target mRNAs was produced and visualized applying Cytoscape software (version 3.8.0).

### 2.6. Cell Growth

Four human OS cell lines, MNNG (Catalogue No.: HTX1631), HOS (Catalogue No.: HTX3087), U2OS (Catalogue No.: HTX1634), and 143B (Catalogue No.: HTX2774), were provided by Otwo Biotech (ShenZhen) Inc. (Shenzhen, China). And one osteoblast cell line named hFOB1.19 (Catalogue No.: CL-0353) that was used as standard control was provided by another company, Procell Life Science&Technology Co., Ltd. (Wuhan, China). All the OS cell lines were incubated with a complete growth medium consisting of Dulbecco's modified Eagle's medium (DMEM, Gibco, Shanghai, China), 10% of fetal bovine serum (FBS, Tianhang, Zhejiang, China), and 1% of dual antibiotics (penicillin and streptomycin) (Solarbio, Beijing, China) in an incubator with the atmosphere condition of humidity and the concentration of carbon dioxide (CO_2_) at 5%; the temperature was set 37°C. At the same time, hFOB1.19 cells were cultured with a particular culture medium for human osteoblast (CM-H111, Procell Life Science & Technology Co., Ltd.) in a cell culture equipment with the atmosphere condition of humidity and the concentration of carbon dioxide (CO_2_) at 5%; the temperature was set at 34°C. And they were passaged with the ratio of 1 : 3 after the cells reached 90% of confluence.

### 2.7. Survival Analysis

The data containing 88 patients suffering from OS was downloaded from an online database, Therapeutically Applicable Research to Generate Effective Treatments (TARGET). And the curve of survival analysis was produced based on the survival time of patients suffering from OS. The Kaplan-Meier plot was adopted to show the probability of survival in the high/low gene expression groups. In the predictive survival curve, the critical value is *p* value < 0.05.

### 2.8. Assay of Quantitative RT-PCR

The total mRNA from cultured cells was purified utilizing the HiPure Total RNA Mini Kit, which was offered by Guangzhou Magen Biotechnology Co., Ltd. (Magen, Guangzhou, China), following the instructions of the manufacturer. Subsequently, the PrimeScript^TM^ RT reagent kit provided by the Takara Biomedical Technology (Beijing) Co. Ltd. (Takara, Beijing, China) was utilized to synthesize the complementary DNA from a certain quality of mRNA (1 *μ*g). The quantitative real-time polymerase chain reaction, hereinafter referred to as qRT-PCR, was then made to assess the expressive level of the key miRNAs or mRNAs in a PCR instrument, Roche LightCycler^®^ 96 SW (Basel, Switzerland), using SYBER green qRT-PCR SuperMix Plus (Roche, 50837000). The cycling reaction procedure was fixed at 95°C for 30 seconds, 45 cycles of 95°C for 10 seconds, followed by 60°C for 60 seconds. The expression of final identified miRNAs or mRNAs was normalized to U6 or GAPDH, respectively, which were employed as intrinsic controls. The expression level of miRNAs or mRNAs was evaluated using the 2^−*Δ*Ct^ comparative method. All qRT-PCR experiments were performed in triplicates. All primers of qRT-PCR used in this research were exhibited in Table 2.

### 2.9. Statistical Analysis

A statistical analysis software (San Diego, CA, USA) named GraphPad Prism 8 was utilized to finish the statistical analysis of data. Statistical differences were computed by one-way analysis of variance using unpaired student tests, and a *p* value less than 0.05 was designated as statistically significant.

## 3. Results

### 3.1. Acquisition of Critical miRNAs and Candidate Genes of miRNAs

To acquire the differentially expressed miRNAs (DE-miRNAs) of the miRNA expression profile dataset (GSE28425), we used a “limma” package in R. According to the following threshold conditions, *p* value < 0.05 and ∣log2(fold − change) | >1, we collected a total of 230 DE-miRNAs, including 114 highly expressed miRNAs and 116 lowly expressed miRNAs in the tumor specimens compared to the normal counterparts. By using the “ggplot2” package in R, all gene expression levels and distribution were shown in a heat map (Figure 2(a)) and a volcano plot (Figure 2(b)), respectively. Next, we obtained the clinical information from the GSE79181 dataset and performed the survival analysis of miRNAs using the “survival” package in R. We acquired 26 miRNAs that are significantly related to the prognosis of OS patients. Among them, 10 miRNAs with high expression in OS patients have poor prognosis (hsa-miR-486-3p, hsa-miR-638, hsa-miR-520c-3p, hsa-miR-320B, hsa-miR-1183, hsa-miR-642, hsa-miR-1255B, hsa-miR-381, hsa-miR-1303, and hsa-miR-221), while 16 miRNAs with low expression in OS patients have poor prognosis (hsa-miR-502-5p, hsa-miR-516-3p, hsa-miR-30a-3p, hsa-miR-888, hsa-miR-520 g, hsa-miR-15b, hsa-miR-107, hsa-miR-99a, hsa-miR-494, hsa-let-7e, hsa-miR-592, hsa-miR-758, hsa-miR-519b-3p, hsa-miR-425, hsa-miR-411, and hsa-miR-374b) (Figure 2(c)). Finally, the high expressed miRNAs with poor prognosis from the GSE79181 dataset were intersected with the upregulated miRNAs in the DE-miRNAs from the GSE28425 dataset (Figure 3(a)). At the same time, the lowly expressed miRNAs with poor prognosis from the GSE79181 dataset were crossed with the downregulated miRNAs in the DE-miRNAs from the GSE28425 dataset. The results showed that only one downregulated miRNA with a poor prognosis, hsa-miR-494, was obtained via the intersection analysis between the GSE79181 and GSE28425 datasets (Figure 3(b)). Through searching the online miRNA database, miRBase, we found that hsa-miR-494 possesses two mature miRNAs: one is hsa-miR-494-5p and another one is hsa-miR-494-3p. Thus, we will focus on analyzing the specific roles of hsa-miR-494-3p and hsa-miR-494-5p in OS for further research.

### 3.2. Enrichment Analyses of GO and KEGG for Target Genes

To earn an in-depth understanding of the downstream outcomes of prognostic miRNA-driven modulation, we predicted the downstream specific targeting factors of hsa-miR-494-5p and hsa-miR-494-3p through four online predictive databases (miRWalk, TargetScan, RNAhybrid, and miRanda). After the intersection analysis of the prediction results of four prediction databases, 2,097 mRNAs were obtained as the particular target mRNAs of hsa-miR-494-3p (Figure 3(c)), and 423 mRNAs were accepted as the particular target mRNAs of hsa-miR-494-5p (Figure 3(d)). To further survey the potential biological meanings of these distinct target genes (2520 mRNAs), we carried out the enrichment analyses of GO and KEGG utilizing a “clusterProfiler” package in R. The result of GO included three varying levels: molecular function, hereafter referred as MF, cell component, hereafter referred as CC, and biological process, hereafter referred as BP. These target mRNAs were mainly enriched in the following biological process relevant to nervous system development, including three significant terms: positive regulation of neurogenesis, gland development, and positive regulation of neuron differentiation. In the CC ontology, the items related to vesicle and nuclear membranes constituted the majority of enriched GO categories, for example, nuclear envelope, cell leading edge, and transport vesicle. The terms of the MF level were significantly associated with the regulation of protein kinase activity, such as DNA-binding transcription repressor activity, nucleoside-triphosphatase regulator activity, and protein serine/threonine kinase activity (Figure 4(a)). Furthermore, the KEGG enrichment data show that MAPK, cAMP, and Ras signaling pathways are the top three enriched KEGG pathways (Figure 4(b)).

### 3.3. Screening of Crucial mRNAs

To distinguish the differentially expressed mRNAs (DE-mRNAs), we downloaded three datasets (GSE16091, GSE16088, and GSE14359) involved in the mRNA expression profile. Due to different technology platforms, different data processing methods often give rise to the systematic nonbiological differences that are commonly referred to as batch effects. Thus, the three datasets on mRNA expression profiles were first merged and normalized to eliminate batch effects using the “SVA” package in R. The boxplots for the three datasets were displayed in Figure 5(a). There is an obvious offset from the overall expression distribution in samples before batch effects removal, indicating the existence of the batch effect. After batch effects removal, the overall expression distribution of the sample was uniform (Figure 5(a)). A total of 12547 genes were obtained from the three datasets. Next, the assay of differential expression on the acquired genes was achieved using the “limma” package in R. We gained 821 DE-mRNAs, including 471 highly expressed and 350 lowly expressed mRNAs under the same screening criteria as miRNA. All gene expression levels and distribution were shown in a heat map (Figure 5(b)) and a volcano plot (Figure 5(c)), respectively. Given that miRNA exerts its biological regulation function mainly through negatively regulating its target mRNAs at the posttranscriptional level, we performed an overlapped analysis by intersecting the upregulated mRNAs in differential expression analysis with the predictive target factors of hsa-miR-494-5p and hsa-miR-494-3p, respectively. These results displayed that 80 upregulated mRNAs were obtained in the mRNAs bound to hsa-miR-494-3p (Figure 6(a)), and 11 upregulated mRNAs were picked up in hsa-miR-494-5p target genes (Figure 6(b)). Finally, a miRNA-mRNA modulation network consisting of hsa-miR-494-5p, hsa-miR-494-3p, and their targeting mRNAs obtained through the intersection was built using Cytoscape software. Interestingly, we found that five mRNAs were shared as common targets of both hsa-miR-494-5p and hsa-miR-494-3p, including Transcriptional Repressor GATA Binding 1 (TRPS1), Tumor Necrosis Factor Superfamily Member 10 (TNFSF10), CD93, SKI Like Proto-Oncogene (SKIL), and Zinc Finger FYVE-Type Containing 16 (ZFYVE16) (Figure 6(c)). These data indicated that hsa-miR-494-5p and hsa-miR-494-3p might have an essential biological effect in the occurrence and progression of OS through modulating these five common target genes.

### 3.4. Survival Analysis and Identification of Key Genes

The prognostic value of five common targeting factors of hsa-miR-494-5p and hsa-miR-494-3p (TNFSF10, CD93, TRPS1, SKIL, and ZFYVE16) was further investigated using survival analysis. The survival analysis results demonstrated that two genes, TNFSF10 and TRPS1, significantly connected with the prognostic value of the patients suffering from OS. Notably, the lowly expressed TNFSF10 was inversely correlated with the excellent outcome of patients suffering from OS, while the highly expressed TRPS1 was positively correlated with the poor outcome of patients suffering from OS (Figures 7(a)–7(e)). Thus, TRPS1 was considered a critical predictive biomarker for predicting patients with OS and may have an important influence on the advancement of OS. Therefore, we established a novel miRNA-mRNA subnetwork consisting of key miRNAs (hsa-miR-494-5p/3p) and their crucial target mRNA (TRPS1) (Figure 7(f)).

### 3.5. Validation of the Expression Level of the Critical miRNAs and mRNAs

To verify the relative abundance of two vital mature miRNAs (hsa-miR-494-5p and hsa-miR-494-3p) and their common target gene, TRSP1, in the human OS cell lines and osteoblasts, we implemented a qRT-PCR analysis. The expression analysis of these critical miRNAs and mRNAs illustrated that contrast to the hFOB1.19 (human osteoblasts), the expression level of hsa-miR-494-3p (Figure 8(a)) and hsa-miR-494-5p (Figure 8(b)) was considerably decreased in HOS, 143B, MNNG, and U2OS cell lines. In contrast, the relative mRNA expression of TRSP1 was considerably augmented in OS cell lines (HOS, 143B, MNNG, and U2OS) in contrast to the hFOB1.19, which is the osteoblasts (Figure 8(c)), confirming a negative correlation between hsa-miR-494-5p and hsa-miR-494-3p and TRPS1. Overall, these data indicated that hsa-miR-494-5p, hsa-miR-494-3p, and TRPS1 could be the candidate prognostic markers and valuable treatment targets for OS.

## 4. Discussion

The etiology and metastatic mechanisms of OS remain unclear, and the rate of long-term survivors in the patients suffering from metastasis or recurrent is still shallow. Many previous investigations based on microarrays have determined the indispensable influence of miRNA in the tumorigenesis and progress of OS [17]. A single miRNA has been proved to modulate target mRNA in various tumor-promoting or tumor-suppressing pathways. However, there are a few reports on the mechanism of the miRNA-mRNA modulation network involved in the initiation and malignant growth of OS. Consequently, to look for novel predictive biomarkers of OS, it is indispensable to explore the modulated mechanisms of miRNA-mRNA interacting network at the system level, which may also help administrate the malignant development of OS.

In this study, we obtained 114 miRNAs that were highly expressed in OS specimens and 116 lowly expressed in OS specimens by analyzing the DE-miRNAs from the GEO database. Importantly, we found that hsa-miR-494 with prognostic significance was significantly downregulated in OS, evidenced by the analysis of survival-significant miRNAs in OS. We further explored the biological functions and canonical pathways of the particular target mRNAs of hsa-miR-494-5p and hsa-miR-494-3p. Importantly, combined with the survival analysis, we found that a critical target gene, TRPS1, was highly expressed in OS patients with poor prognoses. Thus, we generated a miRNA-mRNA regulation subnetwork composed of hsa-miR-494-5p/hsa-miR-494-3p-TRPS1 in OS for the first time.

More and more studies have shown that miRNAs have a negative or positive power on the tumorigenesis and improvement of multiple malignant disorders depending on their distinct downstream target mRNAs. It was previously uncovered that the irregularly expressed hsa-miR-494 is concerned with the tumorigenesis and progress of several types of tumors. Duan et al. [18] provided a piece of evidence that hsa-miR-494 might be a vital regulator in promoting the advancement of nasopharyngeal carcinoma by inhibiting polypeptide N-acetylgalactosaminyltransferase 7 (GALNT7) and cyclin-dependent kinase 16 (CDK16), while hsa-miR-494 has a tumor-suppressing force in ovary carcinoma via suppressing cell migration and growth and promoting cell apoptosis [19, 20]. Zhao et al. [21] revealed that hsa-miR-494 acted as a cancer suppressor against gastric carcinoma. Its expression level in the patients with gastric cancer was notably lesser than that in the control groups. Artificially increasing expression of hsa-miR-494 markedly inhibited gastric carcinoma's growth, migration, and invasion. Similarly, hsa-miR-494 was uncovered to underexpress in oral cancer compared with the matched normal tissues. It also has the inhibition functions on the growing ability of cells by destroying the expression of Homeobox A10 (HOXA10) in oral carcinoma [22]. Moreover, the relative abundance of hsa-miR-494 was drastically lessened in the tissues of cervical intraepithelial lesions compared with normal cervical tissues, and transfection of hsa-miR-494 mimics greatly diminished the proliferation and invasion capability of HeLa cells [23]. Furthermore, compared to the matched normal tissues, the level of hsa-miR-494 was shortened considerably in cancerous tissues of the pancreas. And the pancreatic cancer patients with a lowly expressed hsa-miR-494 have a lower overall survival rate than those with a highly expressed hsa-miR-494 [24]. Moreover, the function of hsa-miR-494 as a tumor inhibitor restricts the proliferation and development of OS. The observably decreased hsa-miR-494-3p was also observed in OS specimens by previous studies [25, 26]. In our work, hsa-miR-494 expression was appreciably suppressed in OS compared with control group, and OS patients with downregulated hsa-miR-494 have a worse prognosis, indicating that our results are consistent with the consequences of previous investigations.

Interestingly, hsa-miR-494 positively regulates the carcinogenesis and progression of tumors also had been observed in numerous malignant illnesses. For example, Xu et al. [27] proved that overexpression of hsa-miR-494 enhances retinoblastoma cells' progression. In addition, the expression of hsa-miR-494-3p had been observed to be observably increased in the tissues of prostate carcinoma. And its expression was positively connected with the level of the specific antigen of the prostate in the patient's serum, indicating that hsa-miR-494-3p is a promising indicator for the diagnosis and treatment of prostatic carcinoma [28]. Thus, these observations combined with our results suggest that hsa-miR-494 exerts two opposite functions depending on the type of tumor. However, most of the previous research is only focused on the tasks of hsa-miR-494-3p, but not implicated in another mature miRNA of pre-miR-494, hsa-miR-494-5p. Our present study illustrated that except for hsa-miR-494-3p, expression of miR-494-5p was remarkably declined in OS cell lines compared with control. Hence, we speculate that hsa-miR-494-5p might synergistically have vital impacts in the progression of OS as well as hsa-miR-494-3p.

In addition, in our study, five mRNAs (TNFSF10, CD93, TRPS1, SKIL, and ZFYVE16) were uncovered as common target factors of both hsa-miR-494-3p and hsa-miR-494-5p. The survival analysis results displayed that only TRPS1 was excessively expressed in OS patients associated with poor outcomes, which is in line with our predicting consequences. Therefore, TRPS1 was determined as a critical downstream target effector of hsa-miR-494-3p and hsa-miR-494-5p and may have pivotal effects in the progression and migration of OS. TRPS1 is a distinctive and atypical GATA family member containing a single GATA-type zinc finger domain [29]. It binds to the GATA sequence and modulates the expression of distinct factors through restraining the transcriptional activity of other GATA regulators [30]. Recent investigations have proved that TRPS1 is commonly overexpressed in several kinds of malignant illnesses, such as breast carcinoma, hepatocellular cancer, prostatic carcinoma, and colon cancer [31–34]. And it is possibly connected with the occurrence, invasion, and distant metastasis of malignant diseases and multidrug-resistance during chemotherapy [35]. Thus, TRPS1 was deemed to be a powerful alternative target for tumor inhibition, and the dysregulation of TRPS1 may be a mechanism involved in tumorigenesis. In recent reports, TRPS1 has been found to positively affect distant metastasis, angiogenesis, and the stage of clinical operation of OS. It can enhance the resistance of multiple chemical medications in the treatment of OS [36]. Consistent with previous studies, our present observations unveiled that the mRNA level of TRPS1 was substantially raised in human OS cells when compared to that in the osteoblast cell line. Therefore, we speculate that TRPS1 may be used as a new cancer marker that provides a reference for judging the prognostic value of patients suffering from OS. However, the regulatory mechanism of TRPS1 in OS and its relationship with miRNA remains to be elucidated. In this research, we uncovered a negative connection between hsa-miR-494-5p/hsa-miR-494-3p and TRPS1, and TRPS1 was predicted to become the common targeting factor of hsa-miR-494-5p/hsa-miR-494-3p by bioinformatics analysis. Therefore, we conclude that two miRNAs, hsa-miR-494-5p and hsa-miR-494-3p, and their common targeting gene, TRPS1, may form a crucial functional axis, which coordinately modulates the activation of protooncogenic signaling pathways that control the occurrence and development of OS.

Though we provided potentially useful biomarkers for diagnosis, prognosis, and therapeutic target of OS and generated a new miRNA-mRNA subnetwork consisting of hsa-miR-494-5p, hsa-miR-494-3p, and TRPS1, there are still some limitations and shortcomings in our research. For example, most of our results were derived from bioinformatics analysis and online prediction databases. The limited number of relevant samples were available for research, and the miRNA-mRNA subnetwork was gained by bioinformatics analysis should be further validated by experiments *in vitro* and *vivo*. Hence, more clinical OS samples should be collected and analyzed, and further in-depth research is needed to apply these potential predictive biomarkers of OS in the clinic.

In summary, we identified two miRNAs, hsa-miR-494-5p and hsa-miR-494-3p, and their common targeting gene, TRPS1, that may have an imperative effect on the progression of OS using bioinformatics methods. And we created a novel miRNA-mRNA interactive subnetwork composed of hsa-miR-494-5p, hsa-miR-494-3p, and TRPS1, extending a deeper understanding of the pathological mechanism of OS. Our data suggest that the miRNA-mRNA functional axis provides valuable clues for exploring potential molecular markers in the prognosis and diagnosis of OS.

## Figures and Tables

**Figure 1:** The workflow of the study. GO: gene ontology; qRT-PCR: quantitative real-time polymerase chain reaction; OS: osteosarcoma; KEGG: Kyoto Encyclopedia of Genes and Genomes; DE: differential expression.

**Figure 2:** Analysis of differentially expressed microRNAs (DE-miRNAs) and survival analysis microRNAs. (a) The DE-miRNAs expression was exhibited through heat map; blue and red indicate low and high expressions, respectively. (b) The all miRNAs expression was exhibited through volcano map. (c) The dendrogram of miRNAs for survival analysis.

**Figure 3:** Prediction of target genes of candidate miRNAs. (a) The intersection of upregulated miRNAs in OS with highly expressed miRNAs that associated with poor prognosis. (b) The intersection of downregulated miRNAs in OS with lowly expressed miRNAs that associated with poor prognosis. (c) The intersection of targeting genes of hsa-miR-494-3p predicted by four prediction tools. (d) The intersection of targeting genes of hsa-miR-494-5p predicted by four prediction tools.

**Figure 4:** Analysis of GO and KEGG. (a) Top 10 GO enrichment annotations of candidate genes; BP, CC, and MF represent the biological process, cell component, and molecular function, respectively. (b) Top 30 signaling pathways in KEGG.

**Figure 5:** Screening for differentially expressed genes (DEGs). (a) Removal of the batch effect; the upper panel represents the sample before batch effect removal, and the lower panel represents the sample after batch effect removal. (b) The heat map of DEGs. (c) The volcano map of DEGs.

**Figure 6:** Screening for candidate mRNAs. (a) The intersection of the targeting mRNAs of hsa-miR-494-3p with highly expressed mRNAs. (b) The intersection of the targeting mRNAs of hsa-miR-494-5p with highly expressed mRNAs. (c) The construction of miRNA-mRNA modulation network consisting of hsa-miR-494-3p, hsa-miR-494-5p, and 86 target mRNAs by Cytoscape.

**Figure 7:** Survival analysis of the cotargeting factors of two key miRNAs. Survival analysis curve of (a) TNFSF10, (b) CD93, (c) TRPS1, (d) SKIL, and (e) ZFYVE16. (f) The miRNA-mRNA regulation subnetwork consisting of hsa-miR-494-3p/hsa-miR-494-5p, and TRPS1 was constructed by Cytoscape.

**Figure 8:** Verification of expression of key miRNAs and mRNAs. The relative expression level of (a) hsa-miR-494-3p and (b) hsa-miR-494-5p was detected in OS cell lines and osteoblasts. (c) The relative mRNA expression of TRPS1 in OS cell lines and osteoblasts. All data were displayed as mean ± SD based on triplicate experiments ^∗∗^*p* < 0.01 and ^∗∗∗^*p* < 0.001.

**Table 1:** Basic information of the microarray datasets.

Data source	RNA type	Platform	Sample number (tumor tissue/normal tissue)
GSE79181	miRNA	GPL15497	25/0
GSE28425	miRNA	GPL8227	19/4
GSE16088	mRNA	GPL96	14/9
GSE14359	mRNA	GPL96	10/2
GSE16091	mRNA	GPL96	34/0
TARGET_OS	mRNA	TARGET	88/0

**Table 2:** List of primer sequences used for qRT-PCR analysis.

Gene	Sequence (5′ to 3′)
Universal U6 primer F (microRNA)	AACGAGACGACGACAGAC
Universal PCR primer R (microRNA)	GCAAATTCGTGAAGCGTTCCATA
GAPDH-F	CCACTCCTCCACCTTTGAC
GAPDH-R	ACCCTGTTGCTGTAGCCA
hsa-miR-494-3p	AGGTTGTCCGTGTTGTCTTCTCT
hsa-miR-494-5p	TGAAACATACACGGGAAACCTC
TRPS1-F	GCTGTCTTCCACGGCTTCTTCTC
TRPS1-R	GCTGCTGCTCTGACACGAAGG

## Data Availability

All data used to support the findings of this study are included within the article.
